The article "The Use of Chest Radiographs and Machine Learning Model for the Rapid Detection of Pneumonitis in Pediatric" was retracted in 2023. Reasons: unreliable results or conclusions; concerns about the data; concerns about the peer review; concerns about the citations.

# The Use of Chest Radiographs and Machine Learning Model for the Rapid Detection of Pneumonitis in Pediatric

**DOI:** 10.1155/2022/5260231

**Published:** 2022-07-21

**Authors:** Khalaf Alshamrani, Hassan A. Alshamrani, Abdullah A. Asiri, F. F. Alqahtani, Walid Theib Mohammad, Ali H. Alshehri

**Affiliations:** ^1^Radiological Sciences Department, College of Applied Medical Sciences, Najran University, Saudi Arabia; ^2^Al-Hussein Bin Talal University, Princess Aisha Bint Al Hussein College for Nursing and Health Sciences, Jordan

## Abstract

Pneumonia is a common lung disease that is the leading cause of death worldwide. It primarily affects children, accounting for 18% of all deaths in children under the age of five, the elderly, and patients with other diseases. There is a variety of imaging diagnosis techniques available today. While many of them are becoming more accurate, chest radiographs are still the most common method for detecting pulmonary infections due to cost and speed. A convolutional neural network (CNN) model has been developed to classify chest X-rays in JPEG format into normal, bacterial pneumonia, and viral pneumonia. The model was trained using data from an open Kaggle database. The data augmentation technique was used to improve the model's performance. A web application built with NextJS and hosted on AWS has also been designed. The model that was optimized using the data augmentation technique had slightly better precision than the original model. This model was used to create a web application that can process an image and provide a prediction to the user. A classification model was developed that generates a prediction with 78 percent accuracy. The precision of this calculation could be improved by increasing the epoch, among other subjects. With the help of artificial intelligence, this research study was aimed at demonstrating to the general public that deep-learning models can be created to assist health professionals in the early detection of pneumonia.

## 1. Introduction

Pneumonia is a serious infection that affects the lungs and is caused by an acute respiratory infection. Inflammation of the lung sacs is usually caused by one of two pathogens: bacteria or viruses [1]. A common lung disease is the leading cause of death worldwide, affecting primarily children (18% of deaths in children under the age of five), the elderly, and patients with other diseases [2, 3]. Although the initial bacterial and viral pneumonia symptoms are similar, the treatment for each is very different. There are various imaging diagnosis techniques available today. While many of them are becoming more accurate, they are also very expensive and inaccessible to most populations or regions. Furthermore, [3] highlights the “shortage of radiology experts in low-resource countries or rural areas” or the “endless waiting lists for diagnoses in certain areas,” which leads to an increase in the severity of the disease and, as a result, its mortality rate [2]. And while diagnostic radiography is the cheapest diagnostic technique, it is also the least ionizing and faster to apply than other techniques. However, the opacities that can be visualized can cause the analyst to misinterpret the results [4]. Many of the studies cited in the bibliographic references section develop machine learning techniques based on deep learning models (hereinafter, deep learning) such as convolutional neural networks (CNN), as well as diagnostic techniques for high-resolution images such as computed tomography (CT). It describes the development of a deep learning architecture for diagnosing severe cases of pneumonia via chest X-ray. They used a data set from the Radiological Society of North America, emphasizing that the data set they provided to the convolutional neural network is specialised in constitutive zones [5].

The article "The Use of Chest Radiographs and Machine Learning Model for the Rapid Detection of Pneumonitis in Pediatric" was retracted in 2023. Reasons: unreliable results or conclusions; concerns about the data; concerns about the peer review; concerns about the citations.

The goal is to develop a machine learning model that helps minimise diagnostic time and improve diagnostic accuracy with the use of radiographs, taking into account that not all hospitals or health care centres have access to more precise diagnostic techniques, either due to budget or architecture, and that there are differences between different regions of the same country, and with the goal of reaching a larger population faster. This project's data classification (images) will correspond to the data collected [6]. This includes 5,856 JPEG chest X-rays taken on children aged 1 to 5 years old in the Canton region and obtained from the Kaggle and Mendeley database platforms (Guangzhou). This database includes both radiographs with and without pneumonia (normal). This project will be divided into the following phases based on the above information and the study conducted [7].

1. Medical detail analysis phase: the most relevant pulmonary radiological characteristics for the detection of pneumonia will be studied, and the differences between viral and bacterial infection will also be analyzed
2. Image labeling phase: data classification with which it is going to work already has the validation of 3 expert technicians in diagnostic imaging. So, the information obtained in phase 1 will be validated in this phase
3. Processing phase: in this phase, the size of the images and possible treatment of their grayscale will be standardized. There are different studies that have used the CNN learning model. In addition, to pretrain, the model, freely available artificial intelligence (AI) libraries developed with Python can be used, such as TensorFlow. The possibility of learning transfer and open-access AI libraries will be studied [7]
4. Training and testing phase: the chosen deep learning model will be trained in this phase. Its performance will be evaluated and validated with the comparisons of the classifications previously made by the experts [7]
5. Statistical analysis phase: the results obtained will be analyzed to determine the accuracy of the classification. This will help me decide if a model upgrade is needed
6. Information visualization phase: the idea is to bring the classification model closer to the user; for this reason, work will be done to generate a web application that accepts images of chest X-rays in JPEG format and gives a result that is easy to understand for the user

The studies of [3, 7] influenced the method used. They have also influenced the strategies learned in relation to personal problem analysis and resolution. Other methods, such as those described, have chosen to follow a combined radiograph model that we believe can meet expectations.

The article "The Use of Chest Radiographs and Machine Learning Model for the Rapid Detection of Pneumonitis in Pediatric" was retracted in 2023. Reasons: unreliable results or conclusions; concerns about the data; concerns about the peer review; concerns about the citations.

### 1.1. Deep Learning and Chest Radiographs

Chest radiography is a diagnostic tool that can be used for the diagnosis of pulmonary pneumonia since it is considered a “fast” tool (the patient has to be exposed to the test for a short time compared to others), less ionizing than others, and the least expensive [3]. Although the final image that an X-ray can offer, in this case of the chest, is full of opacities, the grays usually correspond to known pulmonary structures. Thanks to the studies of opacities, radiologists are able to determine whether or not there is oedema or infection.

With the evolution of medicine and its convergence with artificial intelligence, deep learning comes to our knowledge. Together with the study of chest X-rays, it poses a very powerful diagnostic support tool [8]. As shown in Figure 1(a), with the “naked” eye, it seems almost impossible to differentiate the different lung structures, and the judgment becomes more complicated when the images in Figure 1 are exposed. Grayish tones can be intuited between the viral and bacterial pneumonia images in relation to the normal radiograph. But the difficulty of this diagnosis is clearly appreciated only at first sight.

Thanks to deep learning tools, image classification models can be proposed that help distinguishes between the different opacities and grays that usually appear in chest X-rays and can analyze in a minimum time all the peculiarities of the image from a previous training with a database that helps the model to be able to create a classification or prediction relationship, something that has been tested with promising results in the consulted bibliography.

The article "The Use of Chest Radiographs and Machine Learning Model for the Rapid Detection of Pneumonitis in Pediatric" was retracted in 2023. Reasons: unreliable results or conclusions; concerns about the data; concerns about the peer review; concerns about the citations.

## 2. Methodology

### 2.1. Data Set

The data used in this project was obtained through a platform with a large number of freely accessible databases and images called Kaggle. Mendeley was also used to access the data published in Kaggle. For this project, the data published [7] consisted of chest X-rays performed on children between 1 and 5 years of age in the Canton region. The data has been published in Kaggle by Paul Mooney, its creation is dated March 22, 2018, and its last update (version 2) was on March 24, 2018.

The 1 GB file contains 5856 images in JPEG format classified into different groups:

- Normal chest X-ray images
- Bacterial pneumonia thoracic X-ray images
- Viral pneumonia thoracic X-ray images

### 2.2. Environment

#### 2.2.1. Work Environment

To carry out this project, Google Collaboratory (“Colab”) has been used, which has allowed the code to be executed through the browser and has been able to avoid the problems of lack of memory that occurred in the MacOS (M1) operating system initially used.

#### 2.2.2. Programming Language

Python was chosen as the programming language for the development of this project. It was chosen because it is a simple language when programming and because it has the TensorFlow tool.

#### 2.2.3. Used Bookstores

The libraries used (Figure 2) in this project have been presented:

### 2.3. Data Environment

The data was stored in Drive1 of the UOC's institutional Google account. In the dataset folder, there are the Train (training), Test (Test), and Val (validation) folders that contain the image subgrouped according to diagnosis: normal, pneumonia bacteria (bacterial pneumonia), and pneumonia virus (viral pneumonia). The general working path was drive/MyDrive/TFM_Raquel_Sauras/datasets/chest_xray.

#### 2.3.1. Data Reconfiguration

As shown in Figure 3, the images were reconfigured to the same smaller size, 64 × 64, and transformed to “RGB” so that each of the images had the same number of channels (3).

#### 2.3.2. Data Classification

The imported data had already been initially grouped as follows:

- Train (training): images classified as training. These are the images initially used to train the [7]

- Test (test): corresponds to the images that are used to test the model in question
- Val (validation) in this folder are the images to evaluate the model

Although initially the data was already regrouped, it was decided not to have the initial validation folder since it only contained images of bacterial pneumonia. A random sample was generated to generate the training (train) and validation (val) subgroups, as can be seen in Figure 4. With this decision, the sample of images that were initially 5,856 remained at 5,840, losing 16 images from the initial validation folder.

The article "The Use of Chest Radiographs and Machine Learning Model for the Rapid Detection of Pneumonitis in Pediatric" was retracted in 2023. Reasons: unreliable results or conclusions; concerns about the data; concerns about the peer review; concerns about the citations.

The data was classified as follows (Figure 5):

To verify that the images had been subclassified according to the parameters, the number of classes found was also shown (Figures 4 and 6).

### 2.4. Creation of the Model

The different articles consulted used the CNN model as a reference model in deep learning to classify images. So, he used this model for the classification of chest X-ray images.

To train the model, the Sequential () function was used, to which three convolutional layers were added through the Conv2D class (16, 32, and 64), and when the data were normalized, the “ReLu” function was used as an activator.

The MaxPooling2D function is responsible for reducing the sample in width and height (2D) at the end of each added layer. Ultimately, the flatten() layer is added.

Finally, the Dense function of the union of the layers, with 128 units, was used as the output layer [9].

### 2.5. Training and Validation of the Model

As shown in Figure 7, the CNN model was generated and was compiled and trained using the model.compile and model.fit functions, respectively, shown in Figure 8.

The accuracy parameters of the model were studied and displayed for further evaluation. The acc and loss functions were used for the precision study, as shown in Figure 9.

### 2.6. Model Improvement

To improve the model, information augmentation function was proposed that consists of rotating the images on the horizontal axis to extract the most information from each layer. With the “prepare” function, the data of the images destined for training will be increased since what interests us is to improve the model as shown in Figure 10.

In addition, the number of “epoch-” parameters that determine the number of times that the algorithm will work with all the training data (Figures 11 and 12) was increased about the initial model, from 20 to 30.

### 2.7. Development of the Web Application

First, the optimized model was saved, as shown in Figure 13. NextJS, a JavaScript framework for easily generating web applications, was used to develop the application.

To use the model, it was saved and TensorFlow serving was used, which generates a REST API to be able to interact with the model. A second component uses Flask that is responsible for converting the image that the user uploads to the format that the TensorFlow serving component understands (array of pixels, resizes the image, etc.).

The communication process between the different components can be seen in Figure 14.

The article "The Use of Chest Radiographs and Machine Learning Model for the Rapid Detection of Pneumonitis in Pediatric" was retracted in 2023. Reasons: unreliable results or conclusions; concerns about the data; concerns about the peer review; concerns about the citations.

### 2.8. Publishing the Web Application

The web page consists of a form that allows the user to upload a JPEG image and obtain a prediction. For the publication of the web application, an own domain was used, and a server in AWS was used. In addition, Docker was used for its publication, both the web and the two APIs were containerized, and the Docker containers were deployed on the AWS instance using Docker compose.

## 3. Results and Discussion

The results obtained are shown below:

### 3.1. Initial Model

The initial model, model 1, had 4173 images (1073 normal, 2024 bacterial, and 1076 viral, as shown in Figure 5) and generated an accuracy of 70% and a percentage of loss that exceeds 80%.

Figure 15 shows the relationship between precision and loss according to groups (training and validation) according to the evolution of the epoch. If we look at the relationship between training accuracy and validation accuracy, they show the same trend until 4 epoch is reached, at which point the curves diverge; for training accuracy, it tends to increase, but the same does not happen for validation accuracy, which decreases. In this same figure, the relationship of the loss between training and validation starts with a similar downward trend until epoch 5, when the validation loss increases again until it exceeds the initial levels. On the other hand, the training loss continues with the downward trend.

The accuracy percentage of the model reached 70.19%, and the loss was 2.6756, as can be seen in Figure 16.

### 3.2. Optimized Model

For the optimized model, we observe that (Figure 17) the relationship between training accuracy and validation accuracy tends to increase as the number of epochs increases. Indeed, they do not follow an identical logarithmic increase since the validation precision presents a more “irregular” trend with more increases and decreases depending on the epoch.

In this same figure, the relationship of the loss between training and validation starts with a similar downward trend maintained until the last epoch. A slight rise is observed from epoch 20 on the validation loss graph.

The accuracy percentage of the optimized model reached 78.37%, and the loss was 0.698, as can be seen in Figure 18.

### 3.3. Web Application

The user can now upload the image in JPEG format if they go to “Tria un fitxer,” which they want to analyze, and when they have it selected, you can press “Send.” Based on the image chosen by the user, the web page returns the prediction.

### 3.4. Discussion

Due to different socioeconomic factors, there is a shortage of radiology professionals in relation to the volume of patients who come to the clinic with pulmonary symptoms.

The article "The Use of Chest Radiographs and Machine Learning Model for the Rapid Detection of Pneumonitis in Pediatric" was retracted in 2023. Reasons: unreliable results or conclusions; concerns about the data; concerns about the peer review; concerns about the citations.

Artificial intelligence was aimed at helping professionals establish a faster and more reliable diagnosis that is related or not to the symptoms presented.

Studies such as those reviewed to carry out this work have been able to design applications with very high precision, although always bearing in mind that a radiology professional would have to validate the prediction [10–16]. In this project, data augmentation methods have been used to obtain a classification model with a precision percentage of 78.37%. The generated classification model offers the user a good classification of the images, distinguishing between normal chest X-ray and pneumonia, but the existing opacities can contribute to generating some errors between the differentiation of bacterial and viral pneumonia. For this reason, some studies propose computed tomography as the most effective method for detecting and differentiation of viral and bacterial pneumonia.

One of the limitations that arose during the project was creating the work environment and the lack of memory of the equipment used and the incompatibility of libraries, but thanks to Google Collaboratory, it was possible to solve it. In addition, it allows us to share the code with other researchers [17–22].

Another limitation of the project carried out is that few epochs have been used compared to the studies consulted. In our case, only 20 epochs have been made for the initial model and 30 for the optimized model. This difference in epochs is due to the lack of adequate equipment to make a model that compiles quickly and efficiently, saving time for the researcher [23–26].

It should also be taken into account that only one type of neural network (CNN) has been worked on, and a single model has been generated, which has been improved. It would have been interesting to make more models and compare them with each other since the time factor has also been a limitation for this work.

## 4. Conclusions

Pneumonia is a prevalent lung disease and one of the main causes of death worldwide, affecting different groups. Due to its characteristics and mortality rate, we can add that to the current global pandemic by SARS-COV-2, there is currently a lot of literature accessible to the public. In this work, it has been possible to develop a web application that allows the user to classify the image of interest according to whether or not there is pneumonia and what type. In general, all the specific objectives set have been achieved, and the minimum precision established in objective, which was 70%, was exceeded. With the completion of the project, and with the large amount of bibliography currently existing in relation to the chosen topic, machine learning models become more important to help our professionals diagnose diseases faster and with fewer resources than with adequate treatment. In time, it can save lives.

The article "The Use of Chest Radiographs and Machine Learning Model for the Rapid Detection of Pneumonitis in Pediatric" was retracted in 2023. Reasons: unreliable results or conclusions; concerns about the data; concerns about the peer review; concerns about the citations.

### 4.1. Future Recommendations

The future lines of work that can be proposed as a result of this project could be the following:

- Improve the model until reaching an accuracy percentage of 95%. It is very important to establish a good differentiation between viral and bacterial pneumonia because, as mentioned above, the treatment differs
- Generate a network of professionals where developed models are shared, and databases are also shared to improve existing models. This would contribute to generating the best possible model and being able to share and implement it in all health centers worldwide
- Improve the web application. It would be interesting that both the appearance and the functionality of it offer the user more information about the image of interest and leave a space for the user to share comments such as symptoms or validation (in the case of being a radiologist) of the generated prediction. This would feed and improve the model and open new research lines
- Implement artificial intelligence in most health centers to support diagnosis, offering training and collaboration with health professionals

## Figures and Tables

**Figure 1:** Chest radiographs: normal, viral pneumonia, and bacterial pneumonia.

**Figure 2:** Programming libraries.

**Figure 3:** Image size configuration script.

**Figure 4:** Script on the classification of images according to groups.

**Figure 5:** Classification of images according to type and group.

**Figure 6:** Script where the data is displayed according to the random subclassification.

**Figure 7:** CNN model script using the Sequential () function.

**Figure 8:** Compilation and training phase.

**Figure 9:** Study of the accuracy of the CNN model.

**Figure 10:** Image rotation to increase information.

**Figure 11:** Graphic representation of the process in a neural network. Relationship between Bach and iterations to visually understand the concept of an epoch.

**Figure 12:** Increased information to improve the model.

**Figure 13:** Script to save the optimized model.

**Figure 14:** Scheme of communication between the different components of the web application development.

**Figure 15:** Evolution of precision and loss compared to “epoch.”

**Figure 16:** Accuracy value generated in the initial model.

**Figure 17:** Evolution of precision and loss compared to “epoch.”

**Figure 18:** Accuracy value generated in the optimized model.

## Data Availability

The data used to support the findings of this study are included within the article.
